# Clinical Study on Electronic Medical Neuroelectric Stimulation Based on the Internet of Things to Treat Epilepsy Patients with Anxiety and Depression

This article has been retracted.

**DOI:** 10.1155/2021/6667309

**Published:** 2021-03-17

**Authors:** Bo Zhang, Weijie Wang, Shenguo Wang, Shaoping Li, Mingchao Liu, Lantian Wang, Caijun Yang

**Affiliations:** Neurosurgery Department, The People's Hospital of Zhaoyuan City, Yantai 264030, Shandong, China

## Abstract

With the continuous development and improvement of the level of medical technology in our country in recent years, the treatment of epilepsy has been constantly updated and developed. Nerve electrical stimulation is considered to be a very effective method for treating epilepsy with anxiety and depression. There are many traditional methods for the treatment of epilepsy. For example, vagus nerve stimulation (VNS) has been applied earlier, and the therapeutic effect has been confirmed, but it will cause serious complications and is easier to be uncomfortable; deep brain stimulation for epilepsy is still in the immature stage, and there is no final conclusion. Therefore, this article proposes a clinical study on the treatment of patients with epilepsy with anxiety and depression based on the electronic medical nerve stimulation of the Internet of Things. First of all, this article uses the literature method to study the causes of epilepsy and previous treatment methods. Then, we designed an experimental study of epilepsy with depression based on the Internet of Things electronic medical neuroelectric stimulation therapy and selected the core quality of life questionnaire, SDS, and SAS as observation indicators. Finally, the comparison of epilepsy symptoms and depression and anxiety between the control group and the observation group before and after treatment was analyzed. The results of the experiment showed that, among the 50 subjects in the study, the observation group that used electrical nerve stimulation therapy had 5 people who stopped seizures after treatment, accounting for 10%, while in the control group of traditional drug treatment methods, after treatment, only one person stopped the seizure, accounting for 2%. In addition, the SAS and SDS scores of the observation group were also lower than those of the control group. Therefore, the use of nerve electrical stimulation to treat epilepsy with anxiety and depression symptoms has better performance and can help patients recover as soon as possible.

## 1. Introduction

Epilepsy is a chronic disease. This disease is prone to recurrence and the treatment time is very long. About 30% of patients cannot effectively control the frequency of attacks even after two or three years of treatment. Traditional oral antiepileptic treatment has long been prone to cause mental and psychological disorders, the most common being depression. The combination of depression and epilepsy makes the patient's condition worse and accelerates the development of the condition, and recurrent seizures will also be a vicious circle.

The traditional treatment for epilepsy often leads to other complications to the patient during treatment, which makes the condition of the patients who is already suffering from epilepsy more severe, while suffering the double physical and psychological whammy. In order to cure the condition of patients with epilepsy as soon as possible and improve their depression and anxiety, this article proposes a clinical study on the treatment of patients with epilepsy with anxiety and depression based on the Internet of Things electronic medical neuroelectric stimulation.

*Background and purpose*. Phantom limb pain (PLP) can cause disability in nearly two-thirds of amputees. Therefore, it is necessary to find an effective and cheap treatment that can be self-managed. In the nondrug treatment of PLP, contralateral limb transcutaneous electrical nerve stimulation (TENS) and mirror image therapy are two promising treatment methods. The purpose of this study was to evaluate and compare the effects of mirror therapy and TENS in the treatment of PLP in amputees. 26 PLP patients agreed to participate. A therapist who is blind to the treatment given uses the Visual Analog Scale (VAS) and Universal Pain Score (UPS) to make a preliminary assessment of pain. The patients were randomly divided into I group and II-TENS group. However, he did not study and compare these two treatments to highlight the advantages of electrical nerve stimulation (Tilak et al.) [1]. There is no consistent safe and effective method to treat trigeminal nerve-mediated head shaking. In affected horses, the trigeminal nerve is sensitive and appears to cause neuropathic pain. Percutaneous electrical nerve stimulation (PENS) therapy is a minimally invasive neuromodulation therapy used to treat neuropathy pain. To determine whether PENS therapy is safe as well as the tolerability and effectiveness of trigeminal nerve-mediated head shaking, seven researchers conducted studies on horses diagnosed with trigeminal nerve-mediated head shaking and current clinical symptoms. All operations are performed on a sedated horse. There is a needle-prick-sized area of skin that is desensitized with a local anesthetic to facilitate the insertion of the probe. Under ultrasound guidance, the disposable PENS probe is placed under the skin adjacent to the nerve and the suborbital foramen on the rostral side. According to human clinical data, nerves are stimulated for 25 minutes in accordance with a scheme of alternating frequency and perception threshold. However, there are too many uncertain factors in the experiment, and the experimental results are yet to be confirmed (Roberts et al.) [2]. Depression and anxiety are more common in patients with epilepsy than in the general population, and they are related to inefficient emotion regulation and decreased quality of life. Unfortunately, these diseases are not always correctly diagnosed or treated. Some studies have shown that electrical skin activity can be used as a marker of depression. Observe the depression, anxiety symptoms, defense mechanism, and response to cognitive stimulation in patients with epilepsy, and perform a comparison with the control group to explore the correlation between anxiety and depression symptoms, defense mechanism, and electrical skin activity. Using the State-Trait Anxiety Scale, the Beck Depression Scale, and the defense style questionnaire for 40 copies, 64 epilepsy patients and 66 individuals in control group were investigated by psychological questionnaires. Use the MindLAB device to measure the electrical skin activity. The results show that, compared with the control group, patients with epilepsy had higher levels of anxiety and depression symptoms. Patients also tended to use neurotic defense mechanisms, which may be related to poor emotional regulation [3]. Patients with epilepsy after cognitive stimulation had lower electrical skin activity. There was no statistically significant correlation between electrical skin activity, anxiety, and depressive symptoms. It is concluded that it is necessary to evaluate the anxiety and depression symptoms and defense mechanisms of patients with epilepsy. However, the authors did not give a clear countermeasure to solve this problem [4].

The innovations of this article are as follows: (1) It combines the qualitative analysis and the quantitative analysis, and the qualitative analysis is fully based on the analysis of data. (2) It combines theoretical research and empirical research and presents in-depth study of the theoretical basis of Internet of Things technology. On top of that, empirical research is carried out in combination with the specific conditions of epilepsy patients. (3) It fully absorbs the results of previous research and improves on this basis to propose a nerve electrical stimulation therapy, which can effectively help patients with epilepsy recover.

## 2. Clinical Research Methods Based on the Internet of Things Electronic Medical Neuroelectric Stimulation to Treat Patients with Epilepsy with Anxiety and Depression

### 2.1. Current Status of Treatment of Epilepsy with Anxiety and Depression

#### 2.1.1. Brief Description of Epilepsy Disease

Epilepsy, commonly known as “horn wind” or “sheep epilepsy,” is a chronic disease in which the sudden abnormal discharge of brain neurons leads to transient brain dysfunction [5]. According to existing studies, the incidence of epilepsy is second only to headaches, and it is the second most common disease in the domestic neurology department [6, 7].

#### 2.1.2. Classification of Epilepsy Diseases

The types of epileptic seizures can be divided into partial seizures, general seizures, and difficult-to-classify seizure types [8]. The so-called partial seizure, also called local seizure, refers to changes in specific symptoms when the seizure begins, and neurons in the cerebral hemisphere are initially activated, including simple partial seizures, complex partial seizures, and second full seizures. In full onset, the initial symptoms and changes in EEG refer to the crisis of “two brain hemispheres simultaneously participating” [9]. Difficult-to-classify seizures generally refer to epilepsy diseases that have not yet been classified or cannot be classified due to imperfect data [10, 11].

#### 2.1.3. Causes of Depression with Epilepsy

The causes of seizures include genetic factors, brain disease factors, or other factors, and the influencing factors are complex and diverse [12]. Ion channels and abnormal ion channels are the basis for the body to stimulate tissue regulation. Changes in that coding gene will affect the action of ion channels and may cause specific genetic diseases [13, 14]. Nowadays, idiopathic epilepsy in many people is thought to be an ion channel disease caused by defective genes encoding defective proteins. Among them, the relationship between sodium, potassium, calcium channels, and epilepsy is relatively clear. The reduction of epilepsy is closely related to neurotransmitting substances. Under normal circumstances, irritating and inhibitory neurotransmitting substances are balanced and the nerve membrane is stable [15]. If there are too many irritating nerve-transmitting substances or too small a blocking agent, the balance of stimulation and inhibition will collapse, and the membrane will become unstable and cause seizures. The electrolyte balance in the abnormal microenvironment of nerve cells is the basis for maintaining the normal stimulation of neurons [16]. Adhesive cells play an important role in maintaining the survival environment of neurons. If stellate cells change their ability to take in glutamate or gamma amino acids, they may cause seizures [17].

In addition, the main reasons that patients with epilepsy are prone to depression are lack of knowledge about epilepsy and discrimination against epilepsy patients in society [18, 19]. This will have an impact on the employment, marriage, and family of patients with epilepsy, resulting in increased side effects, and frequent life activities will lead to a lack of family and social support for patients with epilepsy. If this continues, feelings and psychology will change, resulting in inferiority complex. This is also an important social and family psychological factor in epilepsy patients, causing anxiety and depression [20].

#### 2.1.4. Treatment of Epilepsy

The current treatment of epilepsy includes drug therapy, surgical treatment, and neuromodulation therapy [21].

*(1) Medication*. Currently, the main treatment for epilepsy in our country is medication [22]. The prerequisite for choosing epilepsy drugs is to determine the classification of epilepsy symptoms first and, second, to carefully observe the epilepsy symptoms and then make a reasonable drug choice. For example, if infants and young children do not take pills, not only is using syrup preparations beneficial to the child, but also it makes it easy to manage the dosage. When children choose drugs, they need to pay attention to choosing drugs that will not affect cognitive function, memory, and attention. For pregnant women with epilepsy, it is necessary to pay attention to hormones, sexual desire, female characteristics, pregnancy and reproduction ability, and the effect of antiepileptic drugs on teratogenicity. Traditional antiepileptic drugs (e.g., adrenal glands and phenol babbitt, etc.) have certain clinical effects, but they also have many side effects, such as excessive gum formation, increased hair, high teratogenicity, and excessive effects. It is generally difficult for patients to tolerate these side effects. New antiepileptic drugs (e.g., Lamotrigine, Spaphon, and Questine Vitalizer) not only are clinically effective but also have very low side effects and are easily accepted by patients [23, 24].

Patients need to be checked regularly. Doctors must provide individual treatment for each patient's specific state based on science. Under the guidance, complete cooperation between the parties can achieve satisfactory results [25]. In traditional concepts, there may be such an idea that antiepileptic drugs will cost money and will reduce their intelligence and so forth. This will not only help patients with epilepsy but may also miss the best treatment time due to delays in treatment, leading to intractable epilepsy.

*(2) Surgical Treatment*. After drug treatment, one-third of patients will continue to have seizures. About half of patients will get some improvement after surgery [26]. Surgical treatment is suitable for the following situations: (1) Epilepsy is caused by epilepsy drugs that affect daily work and life. (2) The location of the source of some epilepsy is clear, and the concentration is uniformly restricted. (3) Surgical treatment will not cause serious loss of function.

*(3) Neuromodulation Therapy*. Neuromodulation therapy is a new neuroelectrophysiological method and the most promising treatment for epilepsy [27]. rTMS uses pulsed magnetic fields to adjust the bioelectricity of the cerebral cortex and regulate the state of brain function through brain activity, brain blood flow, and metabolism. Magnetic stimulation therapy can reduce the excitability of the cerebral cortex, reduce the frequency of epileptic seizures and abnormal discharge of EEG improvement, and repair brain damage caused by epilepsy and epilepsy treatment to achieve the purpose. rTMS is effective for many chronic brain diseases such as epilepsy. Drugs and surgical treatments will not cause damage to the human body. These two treatment methods can guarantee the patient's cognitive level to the greatest extent and are extremely safe, have almost no side effects, and will not bring about a large economic burden to the patient's family. Many patients can accept this method [28, 29].

### 2.2. Electronic Medical Nerve Stimulation Therapy

Nerve electrical stimulation therapy is a nondrug therapy that enters the human body through the skin and stimulates peripheral nerves with specific frequency pulse currents, thereby reducing the tissue's susceptibility to harmful stimuli. Scholars at home and abroad have discovered that the mechanism of human rehabilitation is related to the electrical signals in the body, and electrical stimulation therapy can play an important role in pain control by using electrical current characteristics [30]. A large number of experimental studies have shown that electrical stimulation can promote the recovery and regeneration of damaged nerves. The TENS instrument parameters are diverse, including frequency, current intensity, and pulse width, so the settings of different parameters also have different effects on the clinical treatment effect. For different types of epilepsy, determining the best stimulation parameters for clinical use, and so forth [31], the standards are also very important.

#### 2.2.1. Frequency of Stimulation

There are many controversies about the effects of different frequencies on the treatment effect, especially on the pain. Studies have shown that low-frequency TENS may release endogenous opioids for analgesia, and high-frequency TENS with a frequency close to 100 Hz may have an effect by releasing serotonin. Studies have shown that the immediate analgesic effects of TENS with different frequencies are correspondingly different.

#### 2.2.2. Current Intensity

The current intensity is generally selected to cause a significant tremor without causing pain in the patient. Different types of pain use different current intensity, and weak stimulation has a better analgesic effect in relieving chronic inflammatory pain. Studies have shown that it is more appropriate to choose 10–30 mA current intensity in the treatment of epilepsy.

#### 2.2.3. Pulse Width

Pulse width is also a very important factor that affects the effect of epilepsy treatment. When the pulse is <100 *μ*s, the skin sensory threshold rises faster, while the pulse width (>600*μ*s) will activate the pain-transmitting fiber. The clinically selected pulse width needs to be able to selectively stimulate the sensory afferent nerve fiber response, with a wide range in 2–200 *μ*s; research shows that, in the treatment of epilepsy patients, the effect is more significant when the pulse width is 40–75 *μ*s.

#### 2.2.4. Stimulation Site

This article uses electrical stimulation therapy, generally using spiral stimulation electrodes implanted in the patient's body, NVP stimulator, and magnetic block.

Figure 1 shows the inhibitory effect of nerve electrical stimulation therapy on epilepsy.

### 2.3. Internet of Things Technology

The Internet of Things refers to general-purpose terminals and facilities such as sensors [32], mobile terminals, industrial terminal systems, numerical control systems, home smart facilities, and video surveillance systems with “inherent intelligence.” In addition, “external activation” of various assets was equipped with RFID, people, and vehicles equipped with wireless terminals [33]. Smart objects are connected to each other through various remote or wireless cables, which can realize interconnection (M2M). It integrates functions with cloud-based SaaS applications, has a suitable information security mechanism, and provides security control in a private network or Internet environment and even personal real-time monitoring. Through location detection, alarm connection, task indication, project management, remote control, safety protection, remote maintenance, online upgrades, statistical reports, decision support, leadership, and other management service functions to achieve comprehensive management, control, and application of safety and environmental protection, we will use convolutional neural networks to improve IoT RFID wireless sensing technology and capabilities [3].

The input of the model is a matrix made based on the power value of each frequency, containing the time-frequency characteristics of each technology occupying that field frequency. The input to the model can be described as follows:

(1) $$\begin{array}{c} X_{s}=\left[x_{i,j},\cdots ,x_{N,M}\right], \end{array}$$

(2) $$\begin{array}{c} i\in \left[1,N\right],\\ s\in \left[1,S\right]. \end{array}$$

The output of the first convolutional pooling layer is

(3) $$\begin{array}{c} O_{1}=\text{pool}\left(\sigma \left(W_{1}^{v}*X_{s}+b_{1}^{v}\right)\right),\;v\in \left[1,c_{1}\right]. \end{array}$$

In the formula, *c*_1_ is the number of convolution filters in the first layer, where ams is the activation function, and *W* and *b* are the weights and bias parameters used in each layer. The activation function converts the output into a data range that is easy to manage and scale. In addition, the combination of activation functions of layers can simulate very complex nonlinear functions. To this end, The ReLU activation function can be expressed by the following formula:

(4) $$\begin{array}{c} \sigma \left(x\right)=\left\{\begin{array}{cc} x, & \text{if }x>0,\\ 0, & \text{otherwise}. \end{array}\right. \end{array}$$

Therefore, assuming *O*_0_ = *X*_*s*_, the output convolutional layer and pooling layer for the *l*th can be written as

(5) $$\begin{array}{c} O_{l}=\text{pool}\left(\sigma \left(W_{1}^{v}*O_{l-1}+b_{l}^{v}\right)\right),\;v\in \left[1,c_{l}\right],l\in \left[1,L-1\right]. \end{array}$$

The features of the feature extraction process have two characteristics: (a) the frequency-time relationship of the prediction task in the training of the convolution and pooling learning model and (b) the features of the convolutional layer learning and output are connected into a dense vector. The dense vector can be written as

(6) $$\begin{array}{c} O_{f}=f\left(O_{L-1}\right), \end{array}$$

where *f* is a flattened function, which represents the connection process mentioned earlier. Finally, the vector is converted into model output through the fully connected layer. Therefore, the model output can be written as

(7) $$\begin{array}{c} {\hat{y}}_{s}=W_{fu}*\left(f\left(\text{pool}\left(\sigma \left(W_{l}^{v}*O_{l-1}+b_{l}^{v}\right)\right)\right)\right)+b_{fu},\;s\in \left[1,S\right]. \end{array}$$

The CNN optimized classification cross-entropy loss function is used in a hot final output layer to measure the difference between the predicted and actual classes.

(8) $$\begin{array}{c} \text{TotalLoss}=\frac{1}{S}\sum_{s=1}^{S}\left(-\log\left(\Psi_{i}\left({\hat{y}}_{s}\right)\right)\right), \end{array}$$

(9) $$\begin{array}{c} \Psi_{i}\left(\hat{y}\right)=\frac{e^{{\hat{y}}_{i}}}{\sum_{k}e^{{\hat{y}}_{k}}}. \end{array}$$

Put the softmax function in Ψ_*i*_. The *Y*_*i*_ nationality represents the correct coding class of a hot score value.

(10) $$\begin{array}{c} \Theta =\underset{\Theta }{\arg\;\min}\left(\frac{1}{S}\sum_{s=1}^{S}\left(-\log\left(\frac{e^{{\hat{y}}_{si}}}{\sum_{k}e^{{\hat{y}}_{s}k}}\right)\right)\right). \end{array}$$

## 3. A Clinical Research Experiment on the Treatment of Patients with Epilepsy with Anxiety and Depression Based on the Electronic Medical Neuroelectric Stimulation of the Internetof Things

### 3.1. Experimental Research Objects of Electrical Stimulation Therapy Epilepsy Patients

This article selected inpatients in the epilepsy department of a domestic hospital from March 2018 to December 2018 and patients diagnosed with epilepsy with anxiety and depression as the research object. This study preliminarily determined the sample size of each group to be 40–45 cases, and the final sample size was determined to be 100 cases. Each of the control group and the Internet of Things group (observation group) has 50 cases.

### 3.2. Inclusion Criteria

1. All meet the diagnostic criteria and classification scheme of the International Epilepsy Federation in 1981, have a clear consciousness, and are 18–60 years old
2. He was admitted to the hospital for treatment because he was diagnosed with epilepsy with anxiety and depression
3. All experiments were carried out with the informed consent of the patients
4. The experimental subjects do not include patients with mental disabilities and severe liver and kidney dysfunction

According to the order of admission, they were randomly divided into two groups: the control group was treated with traditional medicine, and the observation group was treated with electrical stimulation. There are 50 patients in the two groups. The two groups had no statistically significant differences in age, gender, type of attack, course of disease, and so forth (*P* > 0.05), and they were comparable.

### 3.3. Treatment Methods

The treatment of nerve electrical stimulation is to connect to the pulse generator configuration to generate chronic intermittent low-frequency stimulation electrodes on the nerves. The pulse generator is surgically embedded under the skin of the front wall of the chest wall, and the electrode enters the nerve endings through the incision of the epidermis. The stimulation parameters of the pulse generator can be adjusted and controlled by noninvasive methods such as external remote control equipment. The right side of the heart is rich in nerve fibers. As part of the electrode transplantation for surgery, please choose the left side instead of the right side [34]. If stimulated, it will have a bad effect on the heart.

*Methods*. (1) Before treatment, repeatedly explain to the patient the treatment process and the effect of eliminating worries, improve self-confidence, and strive for successful treatment. (2) On the patient's sleeping platform, place the bandaged tongue depressor in the mouth and let the patient bite and fix it. The handled hands and feet should be properly protected, and the hands and feet should be properly fixed. (3) When treating the upper limbs, in order not to affect the breathing and heart rate and cause an accident, please remove the front end of the lower limbs and do not use one contact point on each limb for treatment. (4) Alternating current generally uses a voltage of 40–60V, and the power is 0.1 seconds. Pulse electric rotating motors generally use 20–40 mA of electric power, and the electric power is 0.1–0.2 seconds. In order to achieve better results, the treatment can be repeated once. In the treatment process, pay attention to verbal prompts. (5) After the patient recovers their function, intensive exercise should be encouraged to establish the result. (6) If the treatment effect is not good, the electric energy can be appropriately increased for treatment after 1 to 2 days. The course of treatment and the effect of treatment need to be recorded in the file.

### 3.4. Observation Indicators

QLQ-C30:30 indicates basic quality of life issues, including physical, functional, cognitive, emotional, and social functions, fatigue, pain, nausea, vomiting and wheezing, insomnia, loss of appetite, constipation, diarrhea, and other functional areas. The scores of the 3 main symptom areas and 6 individual areas have a lot to do with physical conditions. In other words, the higher the score, the worse the situation, and the higher the overall quality of life scores for the 5 functional areas and 1 level, the better the quality of life.

### 3.5. Statistical Methods

The statistical method uses SPSS 22.0 statistical software, the measurement data is expressed as mean ± standard deviation (*x* ± *s*), the comparison of measurement data between groups is by *t*-test, the comparison before and after itself is by paired *t*-test, and the count data is by chi-square test. *P* < 0.05 indicates that the difference is statistically significant.

Figure 2 shows the experimental design of nerve electrical stimulation to treat epilepsy.

## 4. Electronic Medical Neuroelectric Stimulation Based on the Internet of Things to Treat Patients with Epilepsy with Anxiety and Depression

### 4.1. Epilepsy Treatment Based on IoT Electronic Medical Neuroelectric Stimulation

The specific data of the experimental subjects are shown in Table 1. The control group is the traditional method of treating epilepsy patients, and the observation group is the use of electronic medical nerve electrical stimulation to treat epilepsy patients. Among them, the ratio of men to women in the control group was 29:21, and the ratio of men to women in the observation group was 27:23. All the ages fluctuate around 30 years. The seizure types are divided into full-onset and partial-onset types. The course of the disease is divided into less than 1 month, 1–3 months, and more than 3 months.

It can be seen from Table 2 that the parameter settings of the nerve electrical stimulation therapy in this article are reasonable and meet the standard of use. First, determine the location of electrical stimulation to ensure that the right medicine is prescribed; then, during the treatment, the stimulation frequency directly affects the pain sensation, and alternating high and low frequencies can play a good stimulating effect; set the current intensity within the range that the human body can bear. Studies have shown that 10–30 mA is the best; the pulse width is set to 40–75 *μ*s.

It can be seen from Table 3 and Figure 3 that the symptoms of the two groups of patients after different treatments are quite different. The treatment in the control group was traditional drug therapy, and the treatment in the observation group was neuroelectric stimulation therapy in electronic medicine. Regardless of whether it is the control group or the observation group, there are obvious recovery effects before and after treatment, but the degrees of recovery are different. Among the symptoms of epileptic seizures, the probability of the control group before treatment was 100%, and the incidence after drug treatment was reduced to 85%; the incidence of the observation group before treatment was 98.6%, and the incidence after treatment was reduced to 45.7%. This is for epilepsy. It is a very effective treatment for the sick. In terms of anxiety and depression, traditional medications cannot help patients solve this problem but can only relieve the symptoms slightly, but the incidence rate is still 90%; the incidence rate after treatment in the observation group is 47.6%, which effectively reduces anxiety and significant symptoms of depression.

After actual treatment, the incidence of epilepsy in the two groups was significantly reduced, and the frequency of seizures in the observation group was significantly lower than that of the traditional drug treatment group. The experimental results are shown in Table 4. Comparing the two data analysis groups in Figure 4, it is found that the treatment status of patients in the observation group is significantly higher than that of the control group. The incidence of epilepsy in patients in the control group was higher than that in the observation group. The difference is statistically significant (*P* < 0.05).

The 7 individual domains are fatigue, pain, nausea and vomiting, insomnia, loss of appetite, breathing difficulties, and financial difficulties. It can be seen from Table 5 and Figure 5 that the physical fatigue caused by the illness is more serious. Control group and observation group are high, 70.01 points and 71.49 points, respectively, but the observation group's scores after treatment dropped to 36.66 points, which clearly shows that electrical nerve stimulation treatment has a good improvement effect. On the other hand, drug treatments are prone to nausea, vomiting, insomnia, and loss of appetite. The control group did not change much. This indicates that the observation group is beneficial to improve postoperative adverse symptoms.

It can be seen from Table 6 and Figure 6 that the performance of the five functional areas in the QLQ-C30 quality table is poor, but the use of electronic medical nerve stimulation can be effectively improved. For obvious performance in role function and emotional function, the observation group scored 46.29 points for emotional function before treatment and 58.39 points after treatment; the score for role function before treatment was 43.29 points, and after treatment it was 65.32 points, and the score for quality of life also changed from the original 42.34 points. It can be seen from Figure 6 that it increased to 58.89 points, while the score difference in the control group before and after treatment is not obvious enough. Therefore, the use of electronic medical neuroelectric stimulation therapy based on the Internet of Things can effectively treat patients with epilepsy and anxiety and depression [35], and this method can improve emotional function.

### 4.2. Symptoms Anxiety Depression Electronic Medical Treatment of Things Based on Electrical Nerve Stimulation

Self-Rating Depression Scale (SDS) and Self-Rating Anxiety Scale (SAS) are widely used in the study of patients with anxiety and depression. Their reliability and validity are very good, and they can effectively reflect the symptoms of depression. The severity and changes of its severity are used to evaluate the subjective emotions of anxiety patients. Each of SAS and SDS contains 20 elements, and the scores for each element are 1, 2, 3, and 4. After adding points, take the approximate point and multiply it by 1.25 to get the standard point. SAS ≥ 50 points indicates high stress and severe anxiety, and SDS ≥ 53 points indicates severe depression.

Quality of life assessment criteria for patients with epilepsy (QOLIE-31) feet consist of 31 elements, including life satisfaction, seizures, mental health, energy/fatigue, cognitive function, drug problems, social function, and overall health awareness [36]. The higher the score, the higher the patient's quality of life.

The experimental scores of the two groups of patients are shown in Table 7. It can be seen from Table 7 that the differences in the three evaluation systems of the two groups of patients at discharge were not statistically significant (*P* > 0.05). From Figures 7 and 8, it can be seen that the SAS and SDS scores of the two groups of patients 6 months after discharge were lower than those at discharge. The SAS and SDS scores of the observation group were lower than those of the control group. The QOLIE-31 scores of the observation group were higher than those of the control group, and the difference was statistically significant (*P* < 0.05).

## 5. Conclusion

This article is mainly based on the clinical research on the treatment of patients with epilepsy with anxiety and depression based on the Internet of Things electronic medical neuroelectric stimulation. Through in-depth understanding of the inner needs of patients with epilepsy, based on the results of previous research on the treatment of epilepsy, the neuroelectric stimulation method is proposed, which improves the past research deficiencies and can solve clinical problems. Through in-depth study of nerve electrical stimulation therapy, an experimental study based on the Internet of Things electronic medical electrical stimulation for the treatment of patients with epilepsy and anxiety and depression was designed, and SAS, SDS, and the core quality of life questionnaire were selected for indicator observation to analyze the onset of epilepsy patients after treatment and the frequency of anxiety, as well as the improvement of anxiety and depression.

The innovation of this article is as follows: First, it combines the qualitative analysis and the quantitative analysis, and the qualitative analysis is fully based on the analysis of data. Second, it combines theoretical research and empirical research and presents in-depth study of the theoretical basis of Internet of Things technology. On top of that, empirical research is carried out in combination with the specific conditions of epilepsy patients. Third, it fully absorbs the results of previous research and improves on this basis to propose a nerve electrical stimulation therapy, which can effectively help patients with epilepsy recover quickly.

The shortcomings of the study in this article are as follows: First, the number of research objects is too small, and the research data needs to be more objectively verified and treated. Second, the Internet of Things technology is not yet mature in clinical research and needs further improvement and development. Epilepsy treatment has always been a difficult problem in our country's medical research. The new research directions proposed in this article will promote the development of clinical research on epilepsy treatment, jointly help patients with epilepsy get healthier as soon as possible, and contribute to the progress and development of neurology.

## Figures and Tables

**Figure 1:** Inhibitory effect of nerve electrical stimulation on epilepsy.

**Figure 2:** Experimental design of neural electrical stimulation in the treatment of epilepsy.

**Figure 3:** Comparison of related symptoms between the two groups before and after treatment (%).

**Figure 4:** A comparative study of seizure reduction frequency between the observation group and the control group in the actual epilepsy treatment [*n* (%)].

**Figure 5:** Comparison of the scores of 7 individual domains before and after treatment between the two groups.

**Figure 6:** Comparison of scores of five functional domains and overall quality of life scores.

**Figure 7:** Comparison of score differences between the two groups of patients at discharge.

**Figure 8:** Comparison of score differences 6 months after discharge.

**Table 1:** Basic information of experimental subjects.

Group	Number of cases	Gender (case)		Age (years)	Seizure type (cases)			Course of disease (cases)		
		Male	Female		Generalized seizure	Partial seizure	Other	<1 month	1–3 months	>3 months
Control group	50	29	21	30.56 ± 3.18	10	34	6	9	18	23
Observation group	50	27	23	31.28 ± 2.73	12	35	3	10	20	20

**Table 2:** Setting of therapeutic parameters of electroneurotherapy

Parameter items	Parameter setting
Stimulus frequency	Alternation of high frequency and low frequency
Current intensity	10–30 mA
Pulse width	40–75 *μ*s
Stimulating site	In the corresponding neurocutaneous ganglion

**Table 3:** Comparison of related symptoms between the two groups before and after treatment (%).

Symptom	Control group		Observation group	
	Before treatment	After treatment	Before treatment	After treatment

Chest tightness	90.1	70.1	97.6	47.6
Chest pain	72.6	38.5	75.0	22.6
Palpitation	55.1	25.1	67.6	22.6
Shortness of breath	47.6	35.1	45.2	20.1
Anxiety and depression	100.0	90.0	97.6	47.6
Seizures	100.0	85.0	98.6	45.7

**Table 4:** A comparative study of seizure reduction frequency [*n* (%)].

Group	Number of cases	Less than 50% reduction in seizure frequency	50%–80% reduction in seizure frequency	More than 80% reduction in seizure frequency	The attack stopped completely
Observation group	50	15 (30)	9 (18)	6 (12)	5 (10)
Control group	50	12 (24)	5 (10)	3 (6)	1 (2)

**Table 5:** Comparison of the scores of 7 individual domains before and after treatment between the two groups.

Project	Control group		Observation group	
	Before treatment	After treatment	Before treatment	After treatment

Tired	70.01	59.62	71.49	36.66
Pain	48.34	46.11	47.22	45.56
Feel sick and vomit	54.45	50.55	53.34	35.56
Insomnia	56.33	45.56	52.21	17.78
Loss of appetite	46.67	42.10	45.56	18.89
Difficulty in breathing	23.34	18.89	22.22	19.98
Economic difficulties	44.45	42.23	42.23	43.34

**Table 6:** Comparison of scores of five functional domains and overall quality of life scores.

Project	Control group		Observation group	
	Before treatment	After treatment	Before treatment	After treatment

Physical function	46.88	55.77	42.33	57.89
Role function	44.99	60.55	43.29	65.32
Cognitive function	51.83	50.55	50.25	56.37
Emotional function	45.28	57.98	46.29	58.39
Social function	48.34	54.45	49.25	56.78
Overall quality of life score	44.25	56.67	42.34	58.89

**Table 7:** Comparison of SAS, SDS, and QOLIE-31 scores between the two groups at discharge and 6 months after discharge.

Group	Number of cases	SAS	SDS	QOLIE-31
*At discharge*	—			
Control group	50	46.6	50.9	42.7
Observation group	50	45.9	51.5	41.9
*T* value	—	0.695	-0.565	1.589
*P* value	—	>0.05	>0.05	>0.05

*6 months after discharge*	—			
Control group	50	43.3	47.7	45.5
Observation group	50	38.9	40.6	56.7
*T* value	—	6.136	7.913	−26.666
*P* value	—	<0.05	<0.05	<0.05

## Data Availability

No data were used to support this study.
